# Identification of Potential Biomarkers and Biological Pathways in Juvenile Dermatomyositis Based on miRNA-mRNA Network

**DOI:** 10.1155/2019/7814287

**Published:** 2019-12-07

**Authors:** Cheng-Cheng Qiu, Qi-Sheng Su, Shang-Yong Zhu, Ruo-Chuan Liu

**Affiliations:** ^1^Department of Diagnostic Ultrasound, The First Affiliated Hospital of Guangxi Medical University, Nanning, China; ^2^Department of Clinical Laboratory, The First Affiliated Hospital of Guangxi Medical University, Nanning, China

## Abstract

**Objective:**

The aim of this study is to explore the potential pathogenesis of juvenile dermatomyositis by bioinformatics analysis of gene chips, which would screen the hub genes, identify potential biomarkers, and reveal the development mechanism of juvenile dermatomyositis.

**Material and Methods:**

We retrieved juvenile dermatomyositis's original expression microarray data of message RNAs (mRNAs) and microRNAs (miRNAs) from NCBI's Gene Expression Omnibus database (GEO, http://www.ncbi.nlm.nih.gov/geo/); through the R package of limma in Bioconductor, we can screen the differentially expressed miRNAs and mRNAs, and then we further analyzed the predicted target genes by the methods such as Kyoto Encyclopedia of Genes and Genomes (KEGG) pathway enrichment analysis and miRNA-mRNA regulatory network construction and protein-protein interaction (PPI) network using Cytoscape 3.6.1.

**Results:**

Compared with normal juvenile skin tissues, 6 upregulated microRNAs and 5 downregulated microRNAs were identified from 166 downregulated microRNAs and 58 upregulated microRNAs in juvenile dermatomyositis tissues. The enrichment pathways of differentially expressed microRNAs include cell adhesion molecules (CAMs), autoimmune thyroid disease, Type I diabetes mellitus, antigen and presentation, viral myocardium, graft-versus-host disease, and Kaposi sarcoma-associated herpes virus infection. By screening of microRNA-messenger RNA regulatory network and construction of PPI network map, three target miRNAs were identified, namely, miR-193b, miR-199b-5p, and miR-665.

**Conclusion:**

We identified mir-193b, mir-199b-5p, and mir-6653 target miRNAs by exploring the miRNA-mRNA regulation network mechanism related to the pathogenesis of juvenile dermatomyositis, which will be of great significance for further study on the pathogenesis and targeted therapy of juvenile dermatomyositis.

## 1. Introduction

Juvenile dermatomyositis (JDM) is a chronic autoimmune connective tissue disease. Its clinical manifestation is inflammatory myopathy with characteristic skin lesions, like Gottron's papules and heliotrope rash [1–4]. The incidence of JDM is about 1.9–4.1/1,000,000 [5]. The pathogenesis in juvenile is not clear yet, the clinical manifestations of JDM are complex, and its serious cases can even worsen and significantly impact on the prognosis, for example, unspecific clinical course, risk of macrophage activation syndrome, and more in general, chronic systemic inflammation [6, 7]. Therefore, it is urgent to find new diagnostic ideas and new therapies for JDM.

More and more literature indicate that miRNAs play a major role in the occurrence, development, and prognosis of inflammatory myopathy [8]. The latest studies using high-throughput microarray to analyze samples from JDM patients and normal juveniles have given us the opportunity to detect and explore different levels of JDM from genome copy number changes and somatic mutations to transcription levels of gene expression changes and discover the entire molecular landscape of inflammation. Although there have been previous studies involving miRNA-mRNA analysis of JDM, in our knowledge, the regulatory network of miRNAs in JDM has not been constructed.

The purpose of this study is to explore the potential molecular mechanism of JDM and identify effective biomarkers for predicting the pathogenesis of disease and finding target therapy directions in JDM.

## 2. Materials and Methods

### 2.1. Microarray Data

Download miRNAs and expression profile data set of GSE49062 [8] and GSE11971 [9] from the GEO database, the downloaded data were analyzed by R 3.5.2 software. The clinical details of GSE49062 and GSE11971 were listed (Tables 1 and 2). The clinical details of GSE49062 and GSE11971 were included (Tables 1 and 2). As to GSE11971, it only has express miRNAs data from females who had JDM, which includes 19 JDM patients and 4 normal. GSE11971 was included in this study because there were no other data on the expression of microRNAs in JDM.

### 2.2. Screen Differentially Expressed miRNAs and mRNAs

According to the data sets mentioned above, the total data were divided into 2 groups: the JDM group and the normal control group. The R package of limma analysis in R software was used to identify the disorder genes in JDM tissue and normal juvenile skeletal muscle tissue. In order to control the error detection rate, the cutoff standard was set to adj. *P* val < 0.05 and the R package of ggplot 2 were used to draw volcanic maps with a threshold of *P* < 0.05 and select the highest 5% of absolute value of logFc for the next step.

### 2.3. miRNA-mRNA Targeting Relationship Prediction

Differentially expressed miRNAs and mRNAs data were input into microDIP (http://ophid.utoronto.ca/mirDIP/). Minimum confidence was set as high (Top 5%), and the number of sources was set as 1. In this way, we can predict the regulatory relationship between differentially expressed miRNAs and differentially expressed genes.

### 2.4. Pathway Enrichment Analysis

The molecular function was studied by the Kyoto Encyclopedia of Genes and Genomes (KEGG), and KEGG pathway analysis was performed on differentially expressed mRNA by Cytoscape's clueGo plug-in.

### 2.5. Construction of an miRNA-mRNA Regulatory Network

Based on the analysis of differentially expressed miRNAs, differentially expressed mRNAs, and enrichment pathways, Cytoscape was used to visualize the miRNAs-mRNA regulatory network.

## 3. Results

### 3.1. Heterogeneity Test and Preliminary Screening of Differentially Expressed Genes

#### 3.1.1. Heterogeneity Test and Preliminary Screening of Differentially Expressed miRNAs

RMA was used to standardize the data of differentially expressed miRNAs and mRNAs. Then, the limma package of the Bioconductor analysis tool was used to make standardized front-box maps and standardized back-box maps (Figures 1 and 2). A total of 224 differentially expressed miRNAs and 4515 differentially expressed mRNAs were screened. Finally, we selected the top 5% differentially expressed microRNAs and mRNAs by the absolute value of logFc, a total of 11 miRNAs, and 224 differentially expressed mRNAs to perform further analysis.

### 3.2. Functional and Pathway Enrichment Analysis

#### 3.2.1. Differential Expression of mRNAs Function and Pathway Enrichment Analysis

KEGG pathway enrichment analysis of differentially expressed genes was performed with clueGo plug-in of Cytoscape. The *P* value was set to <0.05 when the kappa score was set at or above 0.3. KEGG pathways with significant enrichment of these pathways included allograft rejection, Epstein–Barr virus infection, herpes simplex virus 1 infection, chemokine signaling pathway, and TNF signaling pathway (Table 3). Significantly, differential genes were most abundant in the Allograft rejection pathway (Figure 3).

### 3.3. Analysis of miRNA-mRNA Regulatory Network

The predicted regulatory table of miRNA-mRNA was derived from microDIP, which was constructed based on the interaction between miRNA-mRNA pathways (Figure 4). The number of genes around miRNAs regulation or the number of miRNAs around a surrounding gene was defined as degrees, which represented the center of the miRNA-mRNA regulatory network, and the more important of the network was the greater the degree of its base. Obviously, three miRNAs, which include mir-193b (degree = 76), mir-199b-5p (degree = 50), and mir-665 (degree = 43), are at the core of the regulatory network (Table 4).

### 3.4. Construction of PPI Network

Using STRING database to predict gene interaction, set the minimum required interaction score, high confidence (0.700), downloading the protein interaction relationship and importing Cytoscape software to construct the PPI network (Figure 5) of JDM differentially expressed genes. Many of these differentially expressed genes have high node degrees: MX1 (degree = 28), OAS3 (degree = 27), OAS2 (degree = 27), RSAD2 (degree = 26), IFIT3 (degree = 26), XAF1 (degree = 23), IFI35 (degree = 23), IFIT2 (degree = 23), IFI44L IFIT2 (degree = 23), MX2 (degree = 22), DX58 (degree = 21), and STAT1 (degree = 21); these differentially expressed genes are significantly regulated by differentially expressed miRNAs.

## 4. Discussion

Currently, the computational analysis predicts that miRNAs regulate about 30% of all human genes, and the miRNA-mRNA regulatory network regulates a variety of biological pathways and processes through complex relationships [9]. JDM is an autoimmune connective tissue disease with immunological abnormalities and positive autoantibodies. It has intricate clinical manifestations, so that it is sometimes difficult to cure that [10, 11]. Therefore, if not detected and not treated early in time, JDM would lead to poor prognosis and seriously reduce the quality of life of patients, or even endanger the lives of patients [12–15].

In our study, we used a multistep method to identify the differentially expressed miRNAs and their target genes in JDM from chip data, perform functional and pathway enrichment analysis, and construct a miRNA-mRNA pathway regulatory network. We found that KEGG pathways enriched by differentially expressed genes in JDM, including Allograft rejection, Epstein–Barr virus infection, herpes simplex virus 1 infection, chemokine signaling pathway, and TNF signaling pathway. Obviously, target genes were significantly enriched in allograft rejection. The limitation of this study is that it is currently limited to the theoretical level. To obtain further accurate verification, it depends on the further experimental verification, which will be the direction of our future efforts.

Compared with the expression in JDM skeletal muscle tissues with the expression of normal skeletal muscle tissues, mir-193b and mir-199b-5p were significantly downregulated in JDM, and mir-665 was significantly overexpressed in JDM. With the development of miRNAs therapies, some of them are now in a stage of clinical and preclinical trials, and among them, “miravirsen” was the most developed therapy [16]. There are emerging data from human autoimmune diseases studying miRNAs as novel biomarkers in diagnosing and predicting autoimmune diseases course and response to therapy (Table 5). According to the recent literature, mir-193b, mir-199b-5p, and mir-665 miRNAs are expressed differently in JDM, and cause of their expression in other autoimmune diseases has not been reported yet. Nevertheless, they were also expressed differently in gastric cancer, prostate cancer, lung cancer, and so on [30–32]. JDM always progresses with various manifestations due to its complex pathogenesis, and as a result, it is frequently misdiagnosed. The existing criteria for the diagnosis of disease are unsuitable for the detection of early events in JDM, even insufficient for prediction of aggravations and remissions of established JDM. Therefore, one of the most significant challenges in JDM is the discovery of new biomarkers for early diagnosis and for prediction of the response to medications. Recent studies have revealed dysregulated miRNAs expression during the natural course of JDM, indicating that changes in the miRNA level may lead to the molecular mechanisms of the disease. In this aspect, special attention must be paid to miRNAs, the levels of which were shown to correlate with JDM or could be used for diagnostics in JDM-negative patients.

To date, the regulatory mechanisms of mir-193b, mir-199b-5p, and mir-665 in JDM have not been uncovered. Through KEGG pathway enrichment analysis, these miRNAs may be involved in the regulation of the following pathways: allograft rejection, Epstein–Barr virus infection, herpes simplex virus 1 infection, chemokine signaling pathway, and TNF signaling pathway. However, the potential function of miR-193b, miR-199b-5p, and miR-665 in JDM still remains unknown, and some advantages and limitations of this research should be acknowledged. Compared with microarray data, bioinformatics analysis technology appears as a promising approach, and it has an advantage in that it can help in the molecular understanding of these aspects, as the genes, proteins' interactions, pathways enrich, and miRNA-mRNA networks. This is of great help in the study of the pathophysiological molecular mechanism of JDM.

In conclusion, the future research direction of JDM can start with 3 miRNAs: miR-193b, miR-199b-5p, and miR-665. For more indepth research, we can perfect the clinical information of JDM and expand the sample size of JDM population through clinical follow-up in the next stage, and also we can excavate more biological information of JDM through *in vitro* experiments; finally, establishing a reliable animal model of dermatomyositis will be essential to all research areas of dermatomyositis.

## Figures and Tables

**Figure 1:** Box line diagram and volcano map of differentially expressed miRNAs. (a) Differentially expressed miRNAs data sets were not standardized, (b) after standardization of differentially expressed miRNAs data sets, and (c) volcanic maps for differentially expressing miRNAs. Red dots, significantly upregulated genes. Green dots, significantly downregulated genes. Black dots, nondifferentially expressed genes.

**Figure 2:** Box line diagram and volcano map of differentially expressed mRNAs. (a) Differentially expressed mRNAs data sets were not standardized, (b) after standardization of differentially expressed mRNAs data sets, (c) volcanic maps for differentially expressing mRNAs. Red dots, significantly upregulated miRNAs. Green dots, significantly downregulated miRNAs. Black dots, nondifferentially expressed miRNAs.

**Figure 3:** Function and pathway analysis of differentially expressed mRNAs. (a) Bar chart. (b) Pie chart. (c) Pathway enrichment map.

**Figure 4:** miRNA-mRNA regulatory network. The relationship between 9 key miRNAs and 224 target genes. Rectangles, miRNAs. Circles , genes. Red, overexpression. Blue, downregulation. Yellow, enrichment pathways. Straight lines, the regulatory relationship between miRNAs and genes.

**Figure 5:** JDM's PPI network diagram. The circle represents the gene, and the darker color represents a greater degree. PPI, protein-protein interaction.

**Table 1:** Clinical information of GSE49062 included cases.

Group	*n*	Gender		Age (year)	Tissue source
		Male	Female		
JDM	18	8	10	5.98 ± 0.68	Skeletal muscle
Normal control	6	3	3	12.13 ± 1.55	

JDM, juvenile dermatomyositis; *n*, number of cases.

**Table 2:** Clinical information of GSE11971 included cases.

Group	*n*	Gender		Age (year)	Tissue source
		Male	Female		
JDM	19	0	19	5.31 ± 0.58	Skeletal muscle
Normal	4	0	4	Unavailable	Skeletal muscle

JDM, juvenile dermatomyositis; *n*, number of cases.

**Table 3:** Differential expression of mRNAs enrichment pathway.

Pathway	Gene number	*P* value corrected with Bonferroni	Gene list
Epstein–Barr virus infection	14	0.000006091	CD19, CXCL10, DDX58, HLA-A, HLA-B, HLA-C, HLA-F, HLA-G, IRF9, ISG15, OAS1, OAS2, OAS3, STAT1
Hepatitis C	11	0.000101620	CXCL10, DDX58, IFIT1, IRF9, MX1, OAS1, OAS2, OAS3, RSAD2, STAT1, TLR3
Measles	8	0.004296090	DDX58, IRF9, MX1, OAS1, OAS2, OAS3, STAT1, TNFSF10
Influenza A	14	0.000000839	CCL2, CCL5, CXCL10, DDX58, IRF9, MX1, OAS1, OAS2, OAS3, PYCARD, RSAD2, STAT1, TLR3, TNFSF10
Type I diabetes mellitus	5	0.003325171	HLA-A, HLA-B, HLA-C, HLA-F, HLA-G
Autoimmune thyroid disease	5	0.006558777	HLA-A, HLA-B, HLA-C, HLA-F, HLA-G
Allograft rejection	5	0.002068987	HLA-A, HLA-B, HLA-C, HLA-F, HLA-G
Graft-versus-host disease	5	0.002818762	HLA-A, HLA-B, HLA-C, HLA-F, HLA-G
Viral myocarditis	5	0.008802414	HLA-A, HLA-B, HLA-C, HLA-F, HLA-G

**Table 4:** Target miRNAs and their degrees.

miRNAs	DE	degree
miR-193b-3p	DOWN	76
miR-199b-5p	DOWN	50
miR-665	UP	43
miR-378c	DOWN	16
miR-3182	UP	12
miR-3607-3p	DOWN	11
miR-3202	UP	11
miR-95-3p	DOWN	6
miR-642b-3p	UP	4

DE: differential expression.

**Table 5:** Differentially expressed miRNAs in autoimmune diseases.

Autoimmune diseases	Differentially expressed miRNAs		References
	Upregulation	Downregulation	
Juvenile dermatomyositis	miR-193b, miR-199b-5p	miR-665	—

Multiple sclerosis	miR-186, miR-145, miR-125a-5p, miR-331-3p, miR-146a, miR-362-5p, miR-501-5p, miR-491-5p, miR-142-3p, miR-29b, miR-328, miR-92b, miR-30a, let-7b, miR-425, miR-520a-3p, miR-596, miR-378, miR-29c, miR-20b	miR-20a, miR-211, miR-374a, miR-107, miR-633, miR-93, miR-410, miR-196a, hsa-miR-582-5p, miR-579, miR-1251, miR-363, miR-572, miR-519e, miR-32, miR-15b, miR-580, miR-556-5p, miR-510, miR-663, miR-638, miR-369-3p, miR-208b, miR-200a, miR-126	[17, 18]

Type 1 diabetes	miR-375, miR-152, miR-30a-5p, miR-181a, miR-24, miR-148a, miR-210, miR-27a, miR-29a, miR-26a, miR-27b, miR-25, and miR-200a,	miR-21a and miR-93	[19, 20]

Primary biliary cirrhosis	miR-299-5p, miR-328, miR-371	miR-26a, miR-122a, miR-99a	[21]

Graves' disease	miR-17, miR-155, miR-200a1	miR-146a	[22]

Ulcerative colitis	miR-16, miR-21, miR-23a, miR-24, miR-29a, miR-126, miR-195, and Let-7f	miR-192, miR-375, and miR-422b	[23]

Coeliac disease	miR-182, miR-196a, miR-330, miR-449a, miR-492, miR-500, miR-503, miR-504, miR-644	miR-105, miR-124a, miR-135a, miR-189, miR-202, miR-219, miR-299-5p, miR-323, miR-379, miR-380-5p, miR-409-5p, miR-412, miR-512-3p, miR-566, miR-576, miR-600, miR-614, miR-616, miR-618, miR-631, miR-659, miR-31-5p, miR-192-3p, miR-194-5p, miR-551a, miR-551b-5p, miR-638, and miR-1290	[24, 25]

Addison's disease	miR-181a_1	miR-200a_1, miR- 200a2	[26]

Sjogren's syndrome	miR-146a-5p, miR-107, miR-222-3p, miR-324-3p, miR-18a-3p, miR-151a-3p, miR-107, miR-222-3p, miR-324-3p, miR-18a-3p, miR-151a-3p and others	miR-30b-5p, miR-582-5p, miR-30b-5p, miR-582-5p, and others	[27]

Systemic lupus erythematosus	miR-371b-5p, miR-5100, miR-4642, miR518b, miR-548ap-5p, miR-4762-5p, miR-767-3p, miR-4708-3p, and others	miR-148b-3p, miR-146a-5p, miR-451a, miR-223-3p, miR-1246, miR-21-5p, miR-30e-5p, and others	[28]

Rheumatoid arthritis	miR‐16, miR‐146a/b, miR‐155, miR‐150, miR‐223, miR-125b, miR-125a-5p, miR-146a, miR-146b, miR-203, miR-221, miR-222, and others	miR-34a, miR-34b, miR-124a, miR-125a-3p, miR-363, miR-498, miR-451, and others	[29]

## Data Availability

The data used to support the findings of this study are included in the article.
